The article "Deep Learning and Medical Image Processing Techniques for Diabetic Retinopathy: A Survey of Applications, Challenges, and Future Trends" was published in 2023. Journal: J Healthc Eng.

# Deep Learning and Medical Image Processing Techniques for Diabetic Retinopathy: A Survey of Applications, Challenges, and Future Trends

**DOI:** 10.1155/2023/2728719

**Published:** 2023-02-02

**Authors:** Posham Uppamma, Sweta Bhattacharya

**Affiliations:** School of Information Technology and Engineering, Vellore Institute of Technology University, Vellore 632014, India

## Abstract

Diabetic retinopathy (DR) is a common eye retinal disease that is widely spread all over the world. It leads to the complete loss of vision based on the level of severity. It damages both retinal blood vessels and the eye's microscopic interior layers. To avoid such issues, early detection of DR is essential in association with routine screening methods to discover mild causes in manual initiation. But these diagnostic procedures are extremely difficult and expensive. The unique contributions of the study include the following: first, providing detailed background of the DR disease and the traditional detection techniques. Second, the various imaging techniques and deep learning applications in DR are presented. Third, the different use cases and real-life scenarios are explored relevant to DR detection wherein deep learning techniques have been implemented. The study finally highlights the potential research opportunities for researchers to explore and deliver effective performance results in diabetic retinopathy detection.

## 1. Introduction

DR happens to a person affected by diabetes, and consequently, the eyes get affected. In diabetic patients, irregular blood sugar levels are observed. Generally, glucose in the human body needs to be transformed into some form of energy while performing daily activities. When blood sugar levels exceed their normal control limit, organs such as the retina, heart, nerves, and kidneys begin to suffer. In the presence of high blood sugar levels in the human body, there is a serious risk of eye blood vessels being affected to the point where they become completely obstructed, causing blood leakage, the retinal vessels swell, and even new tiny blood vessels are formed on the eye retina. This is known as hyperglycemia; diabetes is categorized mainly into two types: Type 1 and Type 2 diabetes. Type 1 diabetes is an incurable disease that results from abnormalities in the insulin hormone level, which is responsible for controlling blood glucose levels. The evidence is that Type 1 diabetes reduces the secretion of insulin hormones and hinders the ability of patients to maintain proper glucose levels in the body, leading to multiple health issues. In a Type 2 diabetes situation, the insulin hormone does not function in converting glucose to energy. On the contrary, the human body needs an adequate amount of energy to sustain a healthy and normal life and hence becomes dependent on medication to support the deficiency in the insulin level. In both cases of Type 1 or Type 2, regardless of the blood sugar levels, the patient may be affected by diabetic retinopathy, and furthermore, it may lead to complete loss of eyesight [1].

The initial symptoms of DR include blurred vision and eye floaters, and at an advanced stage, patients can lose complete vision if the disease is chronically sustained for a longer period. This disease is indicated by symptoms of different types of eye retinal lesions. These are comprised of hemorrhages (HM), microaneurysms (MA), hard exudates, and soft exudates. Patients who are afflicted with the illness often fail to avail themselves of early diagnosis by identifying initial symptoms. Hence, it is of utmost importance for a person to ensure an eye examination is conducted at least twice a year to eliminate or proactively avoid disease complications. Considering the disease's severity, diabetic retinopathy is categorized, namely, as one that has a low severity and is recognized at an early stage. On the other hand, PDR is of a higher severity level, being detected at an advanced stage [2].

Various techniques are implemented for the diagnosis of DR at an early stage, and machine learning has predominantly contributed to the same. A subset of artificial intelligence is a machine learning technique implemented to improve the learning experience without human intervention. Deep learning is also a technique that is predominantly used in various types of disease prediction. It is a part of artificial intelligence and machine learning, which contribute to numerous developments in areas such as computer vision techniques, image coloring, image captioning, medical image analysis, drug discovery, neural networks, and even fraud detection systems. In deep learning, large datasets are used on which feature extraction techniques are implemented to identify the most significant attributes, and then various data mining algorithms are implemented to perform data analysis and predictions. These techniques work towards achieving optimized, accurate predictive outcomes without human intervention, and hence, disease predictions become trivial at early stages saving the lives of millions of patients. The following Figure 1 shows the relationship between deep learning, machine learning, and artificial intelligence.

### 1.1. Global Statistics on Diabetic Retinopathy

The American Diabetes Association Position (ADAP) has observed significant improvement in diabetic retinopathy detection and treatment due to the prevalent use of optical coherence tomography and intraretinal pathology. These results enable the evaluation of the thickness of retinal fundus images and generate results about microvascular lesions with enhanced accuracy [3]. The statistical report also validates the fact that diabetic retinopathy is a major public health concern in today's society. The prevalence of diabetes mellitus (DM) since 1980 men's rates have risen by 110 percent, while women's rates have risen by 58 percent, which will further increase by 9 and 7.9 percent globally in 2014. It is estimated that there will be an increase of almost 422 million patients suffering from diabetes worldwide in the next couple of years, which might further increase to almost 629 million by 2045 [4]. Similarly, a computer-aided diagnosis system can be used to reduce the burden on ophthalmologists for performing regular screening procedures. Also, various feature extraction methods, classification techniques, and different algorithms are implemented for the early diagnosis of DR [5].

## 2. Related Works

There exists some of the significant studies which are reviewed in the following sections.

### 2.1. Review of CNN-Based Techniques

CNN is one of the deep learning models which is mainly concentrated on image classification and object identification techniques. The study [6] highlighted that deep learning approaches have a significant impact on the automated detection of diabetic retinopathy in comparison to traditional detection methods as it yielded better accuracy, specificity, and sensitivity. The study examined PDR and NPDR in terms of low, medium, and high levels using the Messidor-2 data source constituting fundus photographs. The IDX-DR X2.1 software was used for implementing CNN (convolutional neural network)-based detection techniques so that microvascular diseases could be easily identified. The authors [7] explained the various severity levels of DR emphasizing DME (diabetic macular edema). A DCNN (deep convolutional neural network) technique was implemented with a clinical scaling system to classify the different stages in disease identification methods when applied to the Digi fundus image dataset from Finland. The grading aspects of retinal images were explored and a measure of the disease's seriousness was identified with sensitivity, specificity, and AUC (area under the curve). The study [8] implemented a hybrid-deep learning method for easy recognition of DR with fundus pictures using the EyePACS dataset from the Kaggle repository. Also, linear-SVM techniques based on convolutional neural networks were used to classify the images, which led to enhanced performance.

The authors in [9] presented a deep learning framework that implemented a CNN model consisting of three different layers to identify the different retinal layers that helped to predict diseases such as DR, drusen, CNV (choroidal neovascularization), and DME. Various preprocessing techniques were applied to get enhanced image quality, and optimization techniques were further implemented to remove unnecessary noise from OCT (optical coherence tomography) images, ensuring that accurate results are generated. The authors in [10] mentioned diabetic retinopathy as being one of the most challenging issues. To detect the level of severity, deep visual features are extracted from the images that are D-color-SIFT (color dense in scale-invariant), and the GLOH (gradient location-orientation histogram technique) was implemented. The selected features from the three image datasets, namely, DIRETDB1 and MESSIDOR-2, are fed into the semisupervised multilayer method. The results are validated using the AUC, sensitivity, and specificity metrics. Similarly, the study [11] presented ultrawide-field fundus photographs that provided detailed imaging of the surface of the retina. The study helped to automatically detect diabetic retinopathy using deep learning algorithms such as the ResNet-34 architecture, consisting of 34 layers that enabled classification. Also, the image segmentation method ETDRS-7SF (early treatment of diabetic retinopathy study-7 standard field) was proposed to achieve enhanced results when validating the output using various metrics. The authors of [12] proposed a pretrained image classification technique using CNN models, namely, AlexNet, VGG-16, and SqueezeNet, for classifying diabetic retinopathy images. The customized 5-layer CNN model was a fully connected neural network classifier, which helped in the easy training of the image datasets, and the ReLU activation function was used to achieve better performance. The existing contributions to various diabetic retinopathy datasets with deep learning approaches are shown in Table 1.

### 2.2. Review of DCNN-Based Techniques

The study in [13] highlighted that a convolutional neural network is a major contributor to image prediction. The study proposed a multistage transfer learning approach for various labeling when applied to relevant datasets. Moreover, an automatic identification of diabetic retinopathy using fundus photographs generated Chen's quadratic kappa score, sensitivity, and specificity. The study in [14] focused on the analysis of microaneurysms at the early stages of DR and DME (diabetic macular edema) identification. A DCNN (deep convolutional neural network) model with a lesion detection algorithm was applied to fundus images. A semantic segmentation method categorized the pictures where ophthalmologists could easily detect the severity levels of proliferative and nonproliferative diabetic retinopathy, ensuring enhanced accuracy and efficiency. The authors in [15] aligned with the similar facts that diabetic retinopathy could be identified using deep learning approaches and they can predict various risk factors in patients. As part of the study, the authors proposed a one-field and three-fieldinception-V3 architecture wherein validation was performed considering data from one eye selected randomly from patient data of two datasets. Finally, an internal validation dataset and an external validation dataset of 3678 and 2345 eyes, respectively, were generated. The model's results were checked with AUC, which produced better results than traditional systems. In [16], the authors presented an entropy-based enhancement technique for refining the features of the images on the imbalanced dataset. This method resulted from an enhanced classification using a hybrid neural network and low computational cost. The deep visual features of DR images are enhanced using graph convolutional networks (GCNs) in association with relation-awarechannel-spatial attention (RACSA). In addition, a modified deer hunting optimization algorithm is employed for extracting optimal features for enhanced classification accuracy [17].

### 2.3. Review of Deep Learning-Based Diabetic Retinopathy Screening in Various Areas

The initial survey is conducted highlighting that most deep learning applications use image processing techniques for DR recognition. The number of individuals affected by the disease is expected to grow rapidly in the next 22 years, especially in developing countries. The WHAGAP (World Health Assembly Global Action Plan) has been intended to diminish this ever-increasing number since its inception in 1990 and is still ongoing. The objective is to identify and report all vision-threatening problems and find ways to eliminate them. The only way to reduce the occurrence of the disease is to initiate early and frequent screening of the disease at an early stage among diabetic patients. The traditional techniques fail to serve the purpose, and ophthalmologists remain unable to detect the severity level. The use of machine learning detects the disease at varying severity levels, reduces the complexities involved in traditional detection systems, and thus helps to save the lives of potential patients having a higher chance of getting affected by the disease [18, 19]. The comparison between the normal eye and the diabetic retinopathy-affected eye is specified in Figure 2.

The present study highlights various information pertinent to different deep-learning approaches utilized for the screening of diabetic retinopathy on both publicly available and real-time datasets. The unique offerings of studies are the following:

- The basic information was relevant to the diabetic retinopathy disease, its types, the cause, and its presence globally which kindles the need to review the different techniques involved in it
- The various imaging techniques and implementations of deep learning procedures for diabetic retinopathy screening are explored
- Recent studies and real-life examples of how image processing can be used to help people with diabetic retinopathy are discussed in detail
- Various datasets are identified, contemporary DL techniques are reviewed, and associated challenges are highlighted acting as scope for future study in this area

### 2.4. Organization of the Study

The information can be organized for this study as follows: Section 2 represents a detailed review of studies conducted relevant to deep learning implementations on diabetic retinopathy.  Section 3 represents the background study on diabetic retinopathy emphasizing on deep learning procedures for medical imaging techniques.  Section 4 provides an exhaustive review of the medical imaging procedures utilizing deep learning approaches for the screening of diabetic retinopathy.  Section 5 highlights DR case studies conducted in diversified locations.  Section 6 consolidates various issues and challenges associated with deep learning implementations for DR. Finally, the conclusions and future directions of research are discussed in Section 7.

## 3. Background Study

### 3.1. Diabetic Retinopathy and Related DL/ML Techniques

DR is an eye retinal disease that is one of the most common chronic diseases all over the world. It usually appears when the person has had diabetes for a long period, which the disease may cause. The major issue is that the disease does not reveal diabetic retinopathy's early signs and symptoms. The disease was classified as low, medium, or rigorous to determine its severity. Numerous researchers have worked to prevent this type of disease complication using various machine learning and deep learning techniques. Deep learning applications incorporating medical imaging techniques have been spotlighted due to their ability to generate effective results. These techniques help in the classification and prediction of diseases without much effort. Also, the CNN architecture enables achieving optimized and enhanced quality outcomes in comparison to traditional disease prediction techniques. According to the authors of [20], DR is one of the most complicated diseases that results in vision problems all over the world. Also, this study concentrated on image quality improvement using a contrast-constrained adaptive histogram equalization model for image segmentation. The image was optimized using a Bayesian optimization technique, and the hyperparameter tuning inception-v4 model improved the evaluation results. Some of the applications of deep learning in various disciplines are specified in Figure 3.

The authors [21] study explained an image classification approach using CLAHE (contrast limited adaptive histogram equalization) and HE (Histogram Equalization) techniques. The study implemented the image screening method using CNN on the MESSIDOR dataset. In [22], the study employed the easy identification of retinal disease using deep learning methods. The image preprocessing procedures reduced the image's dimensions using principal component analysis (PCA) and also eliminated noisy data to produce better results. The fire-fly algorithm and standard scalar strategies were used to normalize the data in the study. The study in [23] proposed a Siamese-like structure with a binocular network on CNN for taking fundus images of the left and right eyes. Those features adapt the transfer learning method for classification and prediction. The study computed the quadratic kappa score as one of the metrics to find accuracy and similarity between histogram matrix prediction and actual images. The study in [24] proposed a convolutional neural network with novel AlexNet, VggNet, GoogleNet, and ResNet models for image classification to automatically recognize a set of fundus images. To enhance the performance of image datasets, hyperparameters and transfer learning techniques are considered. Data standardization and data argumentation methods were implemented to improve the quality of images.

The advancement in CNN architecture addressed the CNN pooling layer's low accuracy issue when specifying image view characteristics. Matrix multiplication, dynamic routing, and squashing functions are shown in CapsNet architecture features on the MESSIDOR dataset for enhanced results [25]. In [26], the study proposed three different neural network models and preprocessing techniques to describe how to classify diabetic retinopathy fundus images. The Fuzzy C-means algorithm trains fundus images without sacrificing image quality and the labels cannot be modified. The authors in [27] focused on retinal image lesions to identify the severity level of the illness. The study explained a lesion localization model and a patch-based technique on a deep neural network for various layers of patches applied, wherein the localization of the red lesions was conducted. The results revealed improvement in AUC level, sensitivity, and specificity metrics. The authors in [28] employed a convolutional neural network-based system that works on an entropy image of a green component for classification. Along with that, the grayscale unsharp-masking (UM) technique of image extraction used greyscale images to improve the performance. In [29], the authors proposed a bag of words model for detecting the level of severity in diabetic retinopathy images on the basic applications of support vector machine and random forest. Various preprocessing methods were included as multiclass classifiers were used to classify various severity levels of the disease. The authors in [30] developed a novel automated-feature approach that worked on a large collection of fundus image datasets. The proposed approach helped in the easy identification of diabetic retinopathy using a computer-aided model integrated with a visual heat map. The study in [31] proposed a new dataset named DDR that was used for fundus image collection. Those images for lesion recognition and segmentation at each level recognized the four stages of lesion detection annotations. The study in [32] presented a deep learning interpretable classifier to organize retinal images into various levels concerning the condition. In this approach, a distribution score was obtained in the last layer of image pixel classification, and the pixelwise score propagation model identified the image visual maps.

The DNN (deep neural network) concentrates on a layered approach for feature extraction methods to compute implicit results. Similarly [33], the authors surveyed different computer vision-related approaches for classification, preprocessing, and feature extraction methods recognizing the irregularities in retinal blood vessels. The study in [34] presented the training and test datasets, and DCNN worked to classify fundus photographs. These outcomes indicated DR and the presence of DME (diabetic macular edema). The authors in [35] proposed to find the severity level of the disease using fundus image classification techniques and an image normalization approach to detect the size and shape of the images. On the basis of the processed images, an inception-v4 algorithm was used to enhance the quality of an image. The study in [36] proposed machine learning algorithms such as SVM, KNN (K-nearest neighbor), and bagged trees applied to diabetic patients' physical health records to easily identify diabetic retinopathy. The model generated a superior level of accuracy using the bagged trees prediction method. The authors in [37] proposed a collective intelligence approach (human + eye) for enhanced results in comparison to the traditional artificial intelligence techniques to find the various categories of diabetic retinopathy. The proposed method used EfficientNetB3, EfficientNetB4, and EfficientNetB5 to improve the accuracy of images that had already been trained. This approach restricts a smaller training dataset due to the variance and amount of data distribution. The study in [38] presented a preprocessing approach and a contrast-limited histogram method to refine the images on a dataset and resulting in high-quality images. A multiclass classifier transfer learning method trained with GoogleNet architecture was used to extract the image features to generate efficient results. The study in [39] proposed automatic diagnosis approaches implemented on retinal images to identify the severity of the disease. In this proposed machine learning algorithm, the inception network architecture is trained and tested on the EYEPACS dataset for classifying the fundus images. These approaches yielded enhanced accuracy results in comparison to the traditional approaches. These deep learning and machine learning models also help to detect and prevent various health-related issues, for example, mental disabilities in humans [40]. The CNN model in [41] is used to identify the patient's condition based on image emotion exposure. Moreover, deep learning methods were used to process biomedical signal information. The prognosis of dermatological diseases and related CNN implementations are discussed in [42]. A summary of the various studies reviewed and discussed in this section is presented in Table 2.

### 3.2. Performance Evaluation of the Reviewed DL/ML Implementations

The various DL/ML techniques used in DR diagnosis are critically reviewed. Each of the implementations were evaluated using commonly used metrics such as accuracy, specificity, sensitivity, precision, recall, and ROC. This section presents a comparative analysis of the performance of these techniques as published in the reviewed study. The section also identifies the limitations of each of the implementations which enable researchers to understand the associated challenges thereby providing ideas for model optimization. The consolidated parametric evaluation for performance analysis is presented in Table 3.

## 4. Significance of Deep Learning Applications Using Medical Imaging Techniques

Applications of deep learning have had a significant impact [43] on medical image analysis over the past few years. These applications have helped ophthalmologists easily detect various eye diseases and identify the severity levels of patient conditions relevant to the disease. The significant applications of deep learning for medical image processing are specified in Figure 4. The study in [44] stated that multiple people were identified as suffering from any eye disease at its initial stages by the ophthalmologists using various types of classification rules and prediction techniques to generate the best results. The study in [45], explained that the layered approach of CNN helped to improve the accuracy of predictions concerned with fundus photographs.

The authors in [46], addressed a convolutional neural network model, which was implemented as an effective way to classify and predict the images in different layers leading to optimized performance. It provided real-time classification techniques to employ deep network features to achieve accurate results. The study in [47] discussed medical imaging processes that were used as an effective way to grade the severity levels using a neural network classifier for fundus images. A multistage classification deep neural network was used in association with a shallow dense layer, being applied to the diabetic retinopathy dataset that generated grading of the disease with enhanced accuracy. The study also implemented a graded equalization method to improve the effectiveness and transparency of the pictures for microaneurysm detection.

### 4.1. Classification Techniques

In image processing, the fundus images are classified using a CAD (computer-aided diagnosis) system by implementing various imaging techniques to achieve early diagnosis and clarity regarding patient health conditions. The previous studies explain several preprocessing procedures for DR-related images and classify the presence of DR in a patient. Studies have implemented various classifiers incorporating CNN layers to predict the disease. Also, multicast lesion detection procedures and modified-CNN applications are implemented on fundus images to classify normal PDR and severe NPDR, thereby generating a PDR histogram, threshold edge values, accuracy, and specificity [48, 49]. The authors in [50] used an automatic screening tool for reducing manual interruption and ensuring the diagnosis of the disease in a shorter time frame. These screening methods are implemented in different datasets to classify and detect the DR grade levels thereby implementing different levels of image-enhancing rules such as normalization and extension of the quality of lesions. These lesions can be classified using image-level descriptors to monitor the patient's condition and grade the level of severity [51]. The study in [52] surveyed various traditional works that were performed using several screening methods for early detection of DR. These screening methods are used for image cropping, rotating, and resizing aspects to find mild variations in retinal vessels that generate optimized outcomes.

Additional approaches for evaluating DR levels at the initial stage include using the visual graphic (VG) method for the classification of images and then the performance is calculated using error-correcting output codes (ECOC) classifier [53]. The study in [54, 55], explained the use of pretrained CNN models with a transfer learning approach for the refinement of images. These models classify images using a support vector machine (SVM) considering publicly available databases. DR detections and lesions identification problems can also be resolved using deep MIL (multiple instance learning) wherein handling of the improper DR lesions is performed using a well-trained framework to achieve enhanced quality The earliest sign of retina disease include the identification of exudates, namely, soft and hard exudates. These exudates were identified in terms of yellow color cotton wool spots using morphological methods involving multiple numbers used for the filtering of the retina lesions. The authors in [56, 57] proposed a training method that efficiently identified the existence of exudates using CNN-based framework. Various studies show how normalizing pixel values for training and testing images can be performed with the help of image-enhancing techniques. In [58], the authors proposed a multilayer deep CNN and SVM classifier method that performed DR segmentation and detection. These retinal images were preprocessed using the gaussian filtering method. This method also explained about ways to find the age-related retinal abnormalities along with DR classification. The authors in [59] presented an optical coherence tomography (OCT) approach using 3D-Markov Gibbs random field (MGRF) for extracting higher-order image features. These image features are applied to each layer of the artificial neural network (ANN) classifier to detect DR disease more accurately.

### 4.2. Detection Techniques

Detection means identifying an object or specific part of important data in images. This mechanism mainly worked on the medical imaging process, identifying the defects, and security of the surveillance system. These approaches are bound with computer vision techniques that computed the human vision system complications. In this scenario, artificial intelligence techniques computed enhanced results in image recognition. When it comes to multiimage recognition methods, machine learning and deep learning mechanisms are effectively performed. The study in [60] proposed the detection of medical images using deep learning applications. This study implemented blood vasculature method to detect the retina blood vessels' position in the affected area on images. These vascular results are used by ophthalmologists to give treatment to patients at early stages. The study in [61], explained the SVM method to detect NPDR. The SVM classifier estimated the disease's severity using around 400 test images from the CHASE dataset. Apart from that, a confusion matrix was used to evaluate the results.

Another study in [62] developed a hybrid machine learning method as a detection tool to identify if a patient has retinopathy or not using retinal images. This technique used multiple instances of learning strategies and feature extraction techniques for the results generated. The study in [63], surveyed the results of numerous studies on diabetic retinopathy disease detection and classification issues. It also reviewed microaneurysms, exudates, hemorrhages, and optic disc disorders and their prognosis details. These were used to create awareness on potential future research studies. The authors in [64] developed a DTL (deep transfer learning) approach to detect the various layers of CNN architecture using the inception-v3 algorithm. These methods divided the network into depths and widths to reduce noisy data for enhanced computation results such as sensitivity and specificity.

The study in [65], proposed an image processing method instead of using lesion segmentation and implemented an image classification method. These approaches helped to identify the retinal lesion patches and classified viable retinal vascular along with encoding the texture of the image with local binary patterns. The study in [66] demonstrated an image recognition system for the neurovascular retinal detection method that used a matching filter and a fuzzy entropy-based technique. This technique employs a gaussian filter to precisely recognize small retinal blood vessels in datasets such as MESSIDOR and DRIVE with precise measurements. The study in [67] proposed toboggan segmentation and the multiagent process that worked on the two-sided segmentation of damaged retinal vessels. These were assessed to enhance the quality of the image using filters such as the gaussian and modified kirsch. The authors in [68] explained retinal images based on color characteristics extraction with an ensemble machine learning approach. In this approach, the image analysis, image cropping, resizing, and removal of irrelevant image data were performed using the data source available from the Kaggle repository. Finally, the improved classification metrics were achieved under the ROC curve. The study in [69] presented a novel transfer learning approach for detecting the exudates in retinal images using ResNet-50, inception-v3, and VGG- 19 techniques. These were trained using a CNN model that had already been trained, and then they were applied to one-Ophtma and DIRETDB1 data sources to get accurate classification results.

### 4.3. Segmentation Techniques

Segmentation is a technique for partitioning images into subgroups or segments to reduce complexities in subsequent processing and analysis. The purpose of segmentation is always to change the orientation of an image so as to evaluate it more easily. Also, it could be used to partition the image into sets of pixels, and each pixel gives a clear contrast. This technique yields a high degree of accuracy and enhanced results. In [70], the study proposed a segmentation method that worked on several tissues in the human brain, facial parts, ears, and eyes easily segmented on the visual Chinese human head (VCH) model. Deep learning-based techniques were used on five separate MRI imaging datasets to identify the disease's consequences. It results achieved enhanced accuracy in comparison to the manual segmentation processes. This technique had limitations and is not suited to very big MRI datasets. In [71], The study described how to predict leaf disease and segment it for easy identification, as well as how to use color transforms to find the affected leaf. This study used a k-means clustering algorithm to categorize disease symptoms and separate them as clusters at various stages. The study in [72], proposed a new wavelet-based image segmentation method that involves transforming input images into different orientations while maintaining the standard pixels needed to detect image alterations. To state a clear representation of the specific item, we used morphological approaches to retain specific image segment frontiers.

The authors in [73] proposed a deep-learning architecture with 2D and 3D images for cardiac function segmentation. In this work, 2D modified U-Net architecture was implemented in CNN models segmented on short-axis MR images, resulting in enhanced performance. The authors in [74] stated that segmentation applications play an important role in medical images and Francis' investigation of iris, biometric, and vein segmentation for real-world problems. Deep learning models used encoder-decoder architecture and pretrained classifiers such as VGG-Net, DenseNet, and ResNet to get information that could be used on a large scale. The study in [75] explained MRI brain tumor images and observed a typical tissue to remove noise. The proposed method concentrated on decreasing the noise from a tumor cell and used image segmentation models such as FSSN (Fernandez-Steel Skew Normal), GMM (Gaussian Mixture Model), and Fuzzy C-means.

### 4.4. Registration Techniques

Image registration is an important aspect of the imaging system because it aids in the completion of certain tasks in medical image processing. In feature and intensity-based classifications, image attributes such as image alignment and different measurements are required to acquire results from the target image. The authors in [76] proposed various image registration frameworks for enhanced outcomes based on picture longitudinal values. This study focused on removing noisy data from retinal vessels for enhanced outcomes using quadratic, lower order, and elastic transformation framework models that eliminate errors. The study in [77] proposed fluorescein angiography (FA) and optical coherence tomography (OCT) methods that were identified as scanning laser ophthalmoscope images for future extraction purposes. The resultant extracted features were highly successful in generating global registration results of the complex blood vessel networks pertinent to retinal images. Also, deformable and intensity-based transformations were implemented to improve the motion magnitude of FA and OCT images.

The study in [78] proposed a supervised multispectral fundus image registration (MSI-R-NET) method by analyzing various levels of blood vessel structures in the retina. It also observed the eye movement of retinal vessels for a short period and worked on image irregularity positions. These multispectral images were forecasted without classification and improved outcomes in the training and testing parts. The retinal vessel complications lead to complete vision loss in adults. The authors in [79] presented a novel volume of interest (VOI) for various levels of OT image registration, which offered superior results in B-spline transformations, utilizing a stochastic gradient descent optimizer. Also, it used the Jacobian determinant transformations expansion on retinal vessels and monitored precise values. The study in [80] mentioned the fact that complete image rotations, intensity, and scaling factors are all key challenges in image registrations. To achieve appropriate image feature augmentation, the feature descriptor statistical properties (FiSP) models were employed to ensure minimal scalability. The resized parameters were regulated efficiently, and the resultant outcomes were superior in comparison to traditional approaches. The authors in [81] focused on enhancing the accuracy of retinal images using the SIFT (scale-invariant feature transform) registration method. This method helped in depicting an image of a higher pixel value without using noise data. The automatic image scalability and image alterations were applied to the FIRE dataset to obtain robust values to enable refined scaling and brightness of images, ensuring enhanced performance.

## 5. Deep Learning Algorithms for Diabetic Retinopathy Diagnosis: Case Studies

### 5.1. Use Case 1: Remote Image Analysis Was Used to Diagnose Diabetic Retinopathy in Mexican Patients

The problem of diabetic retinopathy occurs in young- and middle-aged people. The study in [82] suggested the development of an assistive index framework for identifying diseases that are unlikely to be controlled. This study responded to the immediate demand for AI-based DL methods combined with radiographic imaging technology in Mexico to ensure the rapid expansion of artificial intelligence (AI) methods in diagnosis, prognosis, and the provision of quality medical services. ARIA (automated retinal image analysis) is a basic premise of a web-based resource platform consisting of an image analysis module for referable and nonreferable DR classification. The hospital administration provided high-quality services to eye technicians to check the patient's condition and determine the severity of the illness. Both the ophthalmologists' and the ARIA system's results were used to determine the patient's condition. It is an extreme environment to recognize chronic eye diseases such as glaucoma and the DR diagnosis. It also required more ophthalmologists to meet the extremely high standards.

### 5.2. Use Case 2: Andalusian Reginal Government (Spain) to Develop an Automatic Diagnosis Diabetic Retinopathy Prevention Strategy for the Early Stages

The study in [83] addressed the Andalusian Reginal Government of the health ministry of Spain and established an automatic diagnosis preventive system at the beginning stage of diabetic retinopathy. The study used supervised classification algorithms on 1058 images of 529 diabetic retinopathy patients identified by three eye specialists. These experts were from Huelva's Juan Ramon Jimenez Hospital (JRJHH), Cordoba's NASMC (North Area of Sanitary Management), and Seville's VMUHS (Virgen de Macarena University Hospital) who worked on ground truth image assessments to identify the earliest pace of the disease. The complication of diabetic retinopathy caused blindness in 4–11 percent of Spaniards. To ensure the safety of patients, the researchers used an automatic prescreening method to detect hemorrhages and microaneurysms. This system thus needs to concentrate on all eye-related diseases for diabetes patients.

### 5.3. Use Case 3: Monitoring of Diabetic Retinopathy at the Initial Stage in Chinese Patients-A Case Study

The authors in [84] developed the Triglyceride-Glucose Index (TyG) to analyze the diabetes results in Chinese patients. Diabetic patients were registered in 2018 and evaluated by the endocrinology department of a diabetic eye disease center at China Medical University. The two ocular clinical experts on the team classified the patient's condition as mild, moderate, or severe. This study concentrated on the results of the TyG index, BMI (body mass index), and HbA1 (hemoglobin A1c) to predict the level of diabetic retinopathy in people who have had diabetes for a long time. These advancements will be used in the future to enhance diabetic retinopathy prognosis and detect other eye diseases in diabetic-assisted patients.

### 5.4. Use Case 4: Diabetic Retinopathy Affected Regions in America, China, and India

The authors in [85], highlighted diabetic retinopathy to be the primary reason for blindness in America and 99 percent of cases in India. India and China have over 90 million patients suffering from diabetis which could result in unprecendted number of individuals becoming blind in the next few years unless detected early enough. Aravind Eyecare hospitals provide high-quality ophthalmic care. In this study, WiLDNet (Wifi-based Long Distance Networks) technique was used to communicate with patients in rural locations over the online platform. This system ran a mobile health organization for the people who lived in rural areas, which increased the number of patients with favorable prognoses. In this study, various layers of retinal vascular architecture and the system's overfitting of specific dimensions methods implementations cannot be precise. To address such issues, the organization intended to use a large fundus image dataset to improve its performance.

### 5.5. Use Case 5: Computer-Assisted Screening and Detection System in Europe Countries: A Case Study

In this study in [86], according to the World Health Organization (WHO), approximately 422 million people in low- and middle-income countries suffer from diabetic retinopathy. Many people in Europe struggle with vision impairment which can lead to total blindness as well as eye screening programs for diabetic patients are ineffective. During the COVID-19 pandemic, many patients were diagnosed with telemedicine and internet connectivity to consult doctors via online media sources. To accomplish these methods one should be in online mode to save time which is necessary to raise the number of persons registered to a large extent. In [87], the authors discussed fractional-order filters for edge identification in biomedical imaging technologies. The study employed left-sided and right-sidedfractional-order mask filters to fine-tune the image with whole edges detected without noisy data and the performance evaluation of fundus images on the STARE dataset. This process provides complete noise-free images for disease diagnosis.

In the study in [88], the authors proposed a case study to prevent risk factors in diabetic retinopathy in diabetic patients at Tikur Anbessa hospital. A person suffering from diabetes and related complications fail to maintain the required glucose level in the body. On the contrary, such individuals tend to eat healthy diet which have contrareactions of increased blood pressure level and consequential neovascularization. This study suggested frequent health check-ups and glucose levels were used to identify diabetic retinopathy problems in the early years. The study in [89], described the significant factors for the occurrences of diabetic retinopathy in those who had diabetes recognized in Debre Markos Referral hospital in Northwest Ethiopia. Various patients from this hospital maintained retinal vascular images examined using binary and multiple logistic regression approaches. The primary aim of this study is to prevent the occurrences of this disease and conduct a systematic review of screening methods to maintain a healthy glycaemic level.

## 6. Various Issues, Challenges, and Lessons Learned

### 6.1. Lessons

The processing of medical images in a deep-learning environment ensures accurate results. In this study, various methods stated the performance level in 2D images. It is still an ongoing process to be found in deep learning previous work problems, as shown below:

- Most of the cases in traditional works lacked the high resolution of quality images in larger datasets. As a result, creating a proper dataset that collects images of the required quality is necessary. Those images came from several sources, including public and private, and are combined to yield positive results.
- Improved image enhancement and contrast are needed to detect damaged retinal vessels. Because retinal images are small and noisy, it is difficult to identify the disease in the early stage.
- The lack of standardization in data collecting is one of the most significant issues in medical image analysis. It is vital to remember that as the amount of data available grows, so does the necessity for big datasets to ensure that deep learning models produce realistic results.

### 6.2. Issues and Challenges of Diabetic Retinopathy

The following are the challenges and concerns specific to medical image analysis for deep learning applications in the early screening of diabetic retinopathy:

#### 6.2.1. Limited Real-Time Data for Training

Training a large number of images in deep-learning applications is one of the most challenging tasks. The activity of an image dataset with limited images may be tough to integrate with real-time data from other sources, such as hospitals. Also, it obtained enhanced classification and detection accuracy when working with larger datassets.

#### 6.2.2. For Medical Images Collective DL Architecture

In medical image processing, transfer learning approaches were used to identify object detection and classification to achieve enhanced accuracy. But there are scenarios where these approaches failed to deliver optimal classification accuracy. In such cases, it becomes necessary to retrain the model to achieve enhanced accuracy.

#### 6.2.3. The Process of Incorporating DL Applications and Telemedicine

In rural areas, neither medical nor hospitality resources are available to diagnose health issues, especially eye diseases, for which there are no routine screenings. The integration of telemedicine with cloud data sources enables the use of AI techniques to upload images of the retina.

#### 6.2.4. Pool-Based Data Sampling

In this article, traditional image datasets are usually classified as either deep learning or machine learning models. The main concern is that it uses a large volume of records for DR classification and uses both a large amount of processing capacity and memory.

#### 6.2.5. Low Computational Power and Network Size

Two major factors contributed to the deep learning model's overfitting needs: computational power and network size. An object-based screening model is identified as more comfortable in comparison to the image-based screening method popular in medical image processing that examines hemorrhages and other ocular lesions.

## 7. Conclusion and Future Directions

### 7.1. Conclusion

Deep learning is regarded as an effective technique for offering technical solutions in disease prediction and classification. This study discusses various machine and deep learning techniques for the early diagnosis of diabetic retinopathy. These studies were conducted in various geographical locations wherein various DL applications for medical image processing were implemented in the last century. DL has been used to achieve DR identification solutions employing medical imaging techniques such as classification, detection, segmentation, and registration. But, all these various applications of DL incorporating medical image processing methods require enhancement in accuracy, performance, and reduction in computational cost. This study presents an exhaustive review of the various deep learning and image processing-based techniques and relevant applications of the same in DR detection. It also enlists the challenges identified in the earlier studies, namely, relevant to the availability of real-time data, computational power, network size, and various others. Finally, the study mentions certain recommendations for future scope in research that would enable diabetic retinopathy detection at an early stage. These research detections involved facilitating effective hybridization techniques and the implementation of advanced hyperparameter tuning methods to overcome some of the prominent challenges identified in DR detection using DL techniques.

### 7.2. Future Directions

Deep learning algorithms have gained immense momentum in improving diagnosis in medical imaging systems. The traditional studies are concentrated on CNN models and deep-layered architectures to detect diabetic retinopathy. Furthermore, it specifies the use of the massive amount of data presented on image datasets, which was combined with retinal lesions to design a robust model for effective implementation. Due to the limited number of publicly available datasets, DR diagnosis remains a challenge. The recent advancements in DL have produced promising classification results despite having difficulty identifying the damaged lesions. For example, the study in [90, 91] identified segmented intraretinal variations. Images were classified according to their severity level using the multiclass classification approach. This system performed well on various fundus image datasets and identified the patient's condition. These techniques have promising potential in the detection of different eye disorders, namely, glaucoma and other intraretinal abnormalities.

Another future enhancement is identified DR at very large image datasets such as Messidor and EyePACS. To classify the severity level, this system completely relies on the quality of the images that are presented easily. Those images are retrained using the transfer learning method to detect the lesions easily [92]. To develop a system with minimal configuration, overfitting and computational cost need to be reduced.

To overcome the data argumentation issues mentioned in [93], use of more features on the large dataset need to be analyzed to improve accuracy. Both data preprocessing methods and feature enhancement techniques are combined to design a robust hybrid deep learning model for detecting the DR classification and detection. These methods were used to evaluate the information about different patients. It also provides the best outcomes for DR and other eye-related diseases in further proceedings.

## Figures and Tables

**Figure 1:** Relationship between the AI, ML, and DL.

**Figure 2:** Existence of diabetic retinopathy. Source: https://www.kaggle.com/datasets/sovitrath/diabetic-retinopathy.

**Figure 3:** Deep learning applications in various sectors.

**Figure 4:** Applications of deep learning for various medical image processing.

**Table 1:** Various diabetic retinopathy datasets with deep learning implementations.

Ref.	Dataset	Used method	Outcomes and metrics	Pros and cons	Research challenges
[6]	MESSIDOR-2 fundus image dataset	CNN for deep learning	Accuracy, AUC, sensitivity, and specificity	Pros: (i) Efficient screening of DR Cons: (i) Not cost effective	Diversified image datasets are not considered
[7]	Diabetes image dataset + digi fundus Ltd. from Finland	(i) Deep learning CNN based on five-stage diabetic retinopathy screening (ii) Clinical grading system on macular edema	AUC, sensitivity, and specificity	Pros: (i) Ability to increase size of image without modifying structure Cons: (i) Biased results in image feature grading	Inclusion of high-resolution image data but exclusion of low-resolution image data
[8]	EyePACS dataset	Linear-SVM in VGG-Net	Sensitivity and specificity	Pros: (i) Easier identification of DR Cons: (i) Results lack required satisfaction level	Severity level of the disease is not included
[9]	OCT (optical coherence tomography) images	Three-layered CNN	Accuracy, specificity, sensitivity, precession, recall, *F*1 score, and kappa score	Pros: (i) Efficient ocular structure identification Cons: (i) Exclusion of variable eye structure images in the dataset	(i) Use of OCT images alone in implementation (ii) Exclusion of fundus images
[10]	DIRETDB-1, MESSIDOR-2, and FAZ images dataset	(i) Deep visual features (DVF) + D-color-SIFT GLOH technique (ii) Semisupervised multilayer deep learning algorithm	ROC, sensitivity, specificity, and training errors	Pros: (i) Deep visual features are used for reducing time and image uncertainty problems Cons: (i) Inability to perform multiple image classifications at a time	Inability to classify multiple images at a time
[11]	Ultrawide field fundus photographs from St. Mary's hospital in South Korea	ResNet architecture	Accuracy, AUC, sensitivity, and specificity	Pros: (i) Ease in training of huge retinal surface image dataset Cons: (i) Model dependent on single data source for images collection	Segmentation of the huge retinal surface fails to cover mid and far areas of the retina
[12]	RGB images from public MESSIDOR dataset	CNN models-AlexNet and VGGNet-16 SqueezeNet	Sensitivity, specificity, and accuracy	Pros: (i) Enhanced classification accuracy by the pretrained model Cons: (i) Methodology is much generalized to handle diversified problems	Implementation confined to specific problem, generalized conclusion not appropriate
[13]	IDRID (Indian association of diabetic retinopathy dataset) and MESSIDOR dataset	Shapley additive explanation (SHAP) multistage transfer learning approach, (EfficientNet-B4, B5, and SE-ResNeXt50)	Quadratic weighted Cohen's kappa score, sensitivity, and specificity	Pros: (i) Achievement of decreased variation and improved generalization Cons: (i) Lack of stability	Effective hyperparameter optimization method are not included
[14]	IEEE dataset (IDRID)	Deep-CNN model with lesion detection algorithm	ROC, accuracy, and efficiency	Pros: (i) Minimizes darkness of the retinal lesions Cons: (i) Limitations in the data source	Implementations on larger datasets are not performed
[15]	Two datasets, Eye-PACS and 13 medical centers in Thailand	Inception-V3 architecture with one-field and three-field	AUC including risk factors	Pros: (i) Ability to identify several hazards relevant to DR prognosis Cons: (i) Does not include features relevant to DR risks	Deep learning model lacks efficiency, risk analysis, and is not cost efficient

**Table 2:** Various significant machine and deep learning methods in medical imaging analysis.

Ref.	Dataset	Used method	Outcomes and metrics	Research challenges
[20]	MESSIDOR database	HPTI (hyperparameter tuning inception)-V4 model	Sensitivity, specificity, accuracy, and precision factor	Implementation of different classification are models not included
[21]	MESSIDOR database with 400 images	Histogram equalization and limited adaptive histogram equalization methods	Sensitivity, specificity, accuracy, precision, recall, *F*-score, and G-means	Alternative medical databases are not considered for performance evaluation
[22]	MESSIDOR-2 dataset	Principal component analysis (PCA) with firefly algorithm	Accuracy, precision, recall, sensitivity, and specificity	Not suitable for high-dimensional data in various domains
[23]	EyePACS dataset	CNN-based binocular network with siamese-like structure	Sensitivity, specificity, and quadratic kappa score	Use of limited fundus image data having missing values are collected from same patient
[24]	Dataset with 35126 fundus images from kaggle	Feature transfer learning and hyperparameter tuning method	Accuracy, sensitivity, and specificity	Variable image classification methods are not considered to improve model accuracy
[25]	MESSIDOR dataset	Capsule network architecture	Accuracy	Complete classes of image datasets are not trained in CapsNet
[26]	Dataset has 2000 images from the Kaggle	Fuzzy C-means algorithm	Accuracy	System is not implemented in GPU environment, considered limited data sources
[27]	Standard diabetic retinopathy database (DIARETDB1)	CNN with entropy images grayscale unsharp-masking (UM) method	Accuracy, sensitivity, and specificity	Noninclusion of larger datasets
[28]	Kaggle dataset of 21,123 images	Patch-based DNN	Accuracy, sensitivity, and specificity	Considering distinctive labelling model is costly, use of limited image data
[29]	Dataset has 240 images taken from Kaggle	SVM and random Forest techniques	Accuracy	Alternative image classifier methods are not implemented
[30]	MESSIDOR2 and E-ophtha databases	Data-driven algorithm for deep feature extraction	Sensitivity, specificity, and AUC	Time-consuming and increased sensitivity for dataset with multiple variances
[31]	DDR dataset	Deep neural network algorithms-VGGNet-16, ResNet-18, GoogleNet, and DenseNet-121.	Average precision (AP) and IoU (intersection over union) metrics for each type of lesion identification	Detection and segmentation of fundus image lesions from various perspectives are critical, use of larger image datasets are not considered
[32]	Kaggle repository dataset	Score propagation deep learning model	Sensitivity and specificity performance for lesion recognition	Pixel score identification process is not included
[33]	STARE & DRIVE image dataset	Feature extraction + image segmentation method	Sensitivity and specificity performance for lesion recognition	Hybrid robust DL methods are not included for performance enhancements
[34]	EyePACS-1 and Messidor-1 dataset	Deep-CNN-based model	High sensitivity and specificity	Excludes the possibility of model implementation in clinical environment
[35]	STARE, DIARETDB1, MESSIDOR, DRIVE, STARE, REVIEW, and E-ophtha datasets	Deep CNN model with inception-V4 algorithm	Accuracy, precision, and recall	Data from other domains are not included
[36]	Data collected from patients in central India	PCA (principal component analysis) and linear regression	Accuracy	Larger datasets are not considered
[37]	EyePACS dataset	Gaussian filters and EfficientNet	Kappa score and accuracy	Exclusion of balanced dataset leading to reduced efficiency
[38]	Messidor-1	CLAHE method and CNN + transfer learning approach	Accuracy	Exclusion of minor diseases
[39]	EyePACS dataset	Deep-CNN + inception network	Sensitivity, specificity, accuracy, and precision	Automated image prognosis system is not included

**Table 3:** The performance analysis report of various DR detection techniques.

	Ref.	Methods	Metrics (%)	Performance analysis
CNN-based approaches	[20]	Hyperparameter tuning inception V4 model	Accuracy = 99 Specificity = 98 Sensitivity = 99 Precision = 97	Need employment of versatile classification methods
	[21]	Limited adaptive histogram equalization methods	Accuracy = 97 Specificity = 98 Sensitivity = 94 Precision = 97 *F*1 score = 94 G-Means = 94	Image quality needs to be improvised
	[23]	CNN-based binocular network	Specificity = 82 Sensitivity = 7 Kappa score = 0.824	Availability of limited data leading to biased results
	[25]	Capsule network	Accuracy = 95	Training of limited image features
	[26]	Fuzzy C-means	Accuracy = 98	Inclusion of limited datasets
	[33]	Feature extraction + segmentation methods	Accuracy, precision, and recall evaluated DR severity	Need for robust DL techniques to improve results
	[34]	Deep CNN model	Sensitivity = 91 Specificity = 90	System excluded possibilities implementation in clinical environment
	[35]	Deep CNN with inception-V4 model	Accuracy = 88 Precision = 96 Recall = 94	Information from other domains with plausible impact on results are not included
	[37]	EffectiveNet method	AUC = 0.68 Kappa score = 0.36	Biased results are generated from unbalanced dataset
	[39]	Deep CNN with inception method	Accuracy = 92 Specificity = 94 Sensitivity = 81 Precision = 93	Automated image prognosis method is not implemented

Transfer learning approaches	[24]	Transfer learning approach	Accuracy = 97 Specificity = 95 Sensitivity = 92	Biased classification results
	[38]	CNN with transfer learning	Accuracy = 74	Inability to detect minor diseases

Deep neural network-based approaches	[22]	PCA with firefly algorithm using DNN	Accuracy = 97 Specificity = 95 Sensitivity = 92 Precision = 96 Recall = 96	Low-dimensional data are not considered
	[27]	DNN patch-based approach	Accuracy = 97 Specificity = 95 Sensitivity = 92	Use of limited data leading to enhanced cost
	[30]	Deep feature extraction method	Sensitivity = 94 Specificity = 98 AUC curve = 0.97	High computational cost
	[31]	DNN algorithms	Average precision (AP) = 0.88 IoU (intersection over union) = 0.17	Lack of larger datasets
	[32]	Score propagation method	Sensitivity = 91 Specificity = 90	Image pixel score identification model is not included

Machine learning-based approaches	[29]	SVM and random forest techniques	Accuracy = 90	Enhanced image classifier methods are not implemented
	[36]	PCA with linear regression	Accuracy = 92	Larger datasets are not considered

## Data Availability

The datasets and material used to support the findings of the study can be obtained from the corresponding author upon request.
